The article "Value of Defecography in the Diagnostic and Therapeutic Management of the Modified Wells Procedure for Rectal Prolapse" was retracted in 2023. Reasons: signs of a paper mill; suspected computer-generated content; unreliable results or conclusions; lack of ethics approval or compliance.

# Value of Defecography in the Diagnostic and Therapeutic Management of the Modified Wells Procedure for Rectal Prolapse

**DOI:** 10.1155/2022/2219330

**Published:** 2022-04-10

**Authors:** Yangbin Du, Jinxin Zhu, Hailun Li, Zhiqiang Fu, Zhenyu He

**Affiliations:** Department of General Surgery, The Second Affiliated Hospital of Nanjing Medical University, Nanjing 210000, China

## Abstract

The main aim of this study was to explore the role of defecography in the preoperative diagnosis and postoperative evaluation of rectal prolapse surgery (modified Wells procedure). We collected and summarized the X-ray performance and then analyzed the results of 107 patients with defecatory dysfunction who underwent defecography from January 2020 to March 2021. Furthermore, the preoperative and 6-month postoperative defecography results and clinical symptoms of 25 patients who underwent rectal prolapse surgery (modified Wells procedure) were compared. Results showed that among the 107 patients with defecation dysfunction, women had worse defecography results than men (*P* < 0.01). A total of 25 patients successfully completed the surgery without complications such as infection and intestinal fistula and there was no recurrence at 12 months of follow-up. Compared with the preoperative results, anorectal angle during defecation, the depth of rectocele, and perineal descent were significantly improved after the surgery (*P* < 0.01). Moreover, the patient's feeling of obstructed defecation and incomplete defecation was significantly relieved compared to that before the procedure (*P* < 0.01). In conclusion, defecography can be used to diagnose rectal prolapse preoperatively and evaluate the surgical effect combined with clinical symptoms postoperatively, which provides a clinical reference.

## 1. Introduction

Defecography is a method involving static and dynamic examination of the anorectal region of the patient by radiography during simulated defecation [1]. A previous study concluded that it is a sensitive and better method than traditional barium enema and endoscopy for the diagnosis of rectal prolapse and internal rectal prolapse [2]. It is worth noting that rectal prolapse is a complete prolapse of all layers of the rectum through the anus, usually accompanied by depression of the rectovaginal fossa or rectal bladder fossa, loosening of the connection between the rectum and the sacrum, laxity of the lateral ligaments, relaxation of the anal sphincter, and perineal descent. The diagnosis of internal rectal prolapse is usually radiological, and studies have shown that endorectal prolapse usually begins with intussusception 6 to 8 cm above the anal verge. Under the influence of aging, vaginal delivery, and menopause, the degree of intussusception gradually deepens, and contents of the intussusception gradually change from the initial mucosa to the muscular layer, eventually forming a rectal prolapse. Therefore, endorectal prolapse is considered a precursor of rectal prolapse [3].

Defecography Oxford Grading classifies rectal prolapse and endorectal prolapse into five grades [4]. In general, patients with rectal prolapse (grades V) and severe internal rectal prolapse (grades III-IV) require surgical treatment after the failure of conservative treatment [5]. The current surgical procedures are mainly divided into trans-perineal approach and transabdominal approach. Among them, trans-perineal surgery is less invasive but has a high recurrence rate, whereas transabdominal surgery is more effective and has a lower recurrence rate than trans-perineal surgery [6]. In this study, a laparoscopic modification of the Wells procedure was used, which was proposed by Wells in 1958 and later improved laparoscopically by Himpens and is still widely used in the clinical treatment of rectal prolapse [7]. However, to date, there is only a handful of studies on the efficacy of the laparoscopic-modified Wells procedure assessed by defecography. Herein, defecography was performed on 25 patients who underwent this procedure in the Second Affiliated Hospital of Nanjing Medical University to compare the morphological changes of the anorectum before and after the procedure, evaluate the degree of improvement of patients' symptoms, and investigate the corrective effect of the procedure on the pathological state of the anorectum. It is expected that the findings of this study will provide a theoretical basis for the treatment of rectal prolapse and internal rectal prolapse.

## 2. Materials and Methods

### 2.1. Patients

A total of 107 patients who underwent defecography in the general surgery clinic of the Second Affiliated Hospital of Nanjing Medical University from January 2020 to March 2021 were selected. Among them, nine patients with rectal prolapse (grade V) and 16 patients with severe internal rectal prolapse (grade III-IV) were treated by the modified Wells surgery. Notably, PPH was further performed on 19 patients with rectocele. The 25 patients (9 males and 16 females) enrolled in this study had a mean age of (57.8 ± 10.06) years and a disease duration of (6.24 ± 2.67) years. All patients were operated by the same primary surgeon. The age, gender, disease duration, operation time, bleeding volume, and bowel recovery time of patients were recorded. Notably, this study was approved by the ethics committee of the Second Affiliated Hospital of Nanjing Medical University.

The following inclusion criteria were applied for surgical patients: (1) the imaging diagnosis of rectal prolapse and internal rectal prolapse were based on Oxford radiological grading criteria; (2) had obvious clinical symptoms and failed conservative treatment; (3) preoperative coagulation function, and liver and kidney function tests were normal; (4) no other serious underlying diseases were found; and (5) had the independent behavioral ability and could understand and cooperate with the examination.

In addition, the exclusion criteria were as follows: (1) a history of abdominal or perianal surgery; (2) intestine occupying lesions or inflammatory bowel disease found by colonoscopy; (3) slow transit constipation based on the transit test; and (4) CT or MR showing prolapse of other organs, such as uterine prolapse.

### 2.2. Defecography

To prepare the bowel for defecography, patients were asked to have a rectal cleansing enema at home 3 h prior to the examination. Upon arrival at the hospital, the radiologist clearly explained the procedure and precautions to the patient to reduce anxiety and obtain the patient's cooperation. Next, the patient was placed in the left lateral position, and then 400 ml of barium paste (75% w/v barium sulfate) was injected into the rectum via a lubricated enema head. Ortho- and bilateral oblique radiographs were taken in the supine position. The test table was then tilted upright, and the patient was asked to sit sideways on a portable transilluminated toilet. Serial X-rays were taken while resting, squeezing, and excreting rectal contents. Notably, patients were not asked to perform the Valsalva maneuver because some of them had symptoms of fecal incontinence. The total time for the procedure was approximately 10 min.

All patients were examined by the same group of radiologists preoperatively and 6 months postoperatively. All defecography images were analyzed by a radiologist with 30 years of experience and were defined in accordance with the study by Pomerri et al. [8].

### 2.3. Modified Wells Procedure

Preoperative bowel preparation was first performed. All patients underwent the procedure in a modified lithotomy position using stirrups to abduct the legs and limit hip flexion. After entering the abdomen, an initial examination is performed. If the patient was female, the uterus would be suspended by a stitch. The rectum is then grasped and elevated and the right peritoneal reflex of the rectal mesentery is opened with an ultrasound knife. Next, the rectovaginal septum and posterior rectal mesentery are accurately separated without separating the lateral ligaments, thereby moving the rectum.

A polypropylene mesh (10 × 6 cm) is then secured to the sacrococcygeal region. The lateral-free edge of the patch is then sutured to the lateral wall of the rectum with a nonabsorbable suture. After observing the pelvis again, the pneumoperitoneum is closed, the laparoscopic instruments are removed, and the incision is sutured.

Rectal palpation is performed again after abdominal surgery. PPH is performed in patients with rectocele. After the circular anal canal dilator is inserted into the anal canal and fixed to the perianal skin, a purse-string suture is used 3-4 cm above the dentate line. The anastomosis is placed in front of the yellow circle by fixing a circular mucosal suture around the central bar of the anastomosis. The anastomosis is then closed and fired, thereby removing the rectal mucosal band in the process. For women, the vagina is palpated prior to firing to ensure that it is not included in the resection.

All patients are allowed fluid supplementation postoperatively, and the discharge criteria included tolerance of three solid meals and bowel movements.

### 2.4. Statistical Analyses

All statistical analyses were performed using SPSS (version 25.0) statistical software. Measurement data were expressed as mean ± SD, whereas the classified data were represented by a case number. The defecography indexes of patients before and after surgery were compared using paired *t*-test, chi-square test, Fisher's exact test, and McNemar's test. *P* < 0.05 was considered statistically significant.

## 3. Results

For patients who visited the general surgery clinic of the Second Affiliated Hospital of Nanjing Medical University since January 2020, the receiving physicians suggested that patients undergo defecography based on the patients' anal palpation and the patients' feeling of obstruction and incomplete defecation. Consequently, a total of 107 patients had undergone defecography between January 2020 and March 2021, including 63 females and 44 males. A significantly higher proportion of female patients had severe endorectal prolapse, and a significantly higher proportion of combined rectal protrusion and perineal descent compared to male patients (*P* < 0.01). However, there were no significant differences in the rates of spastic pelvic floor syndrome, colonic redundancy, and sacrorectal separation as shown in Table 1.

Patients with rectal prolapse and endorectal prolapse were frequently associated with perineal descent and rectocele. The proportion of patients with rectal prolapse and severe internal rectal prolapse combined with perineal descent was significantly higher than that of patients with mild endorectal prolapse (88.33% vs 41.67%, *P* < 0.01). In contrast, the proportion of patients with mild endorectal prolapse combined with spastic pelvic floor syndrome was higher (*P* < 0.01). Otherwise, there was no significant difference in the proportion of patients with combined rectocele and colonic redundancy as shown in Table 2.

Among the 107 patients who underwent defecography, nine had rectal prolapse (grade V) and 16 had severe internal rectal prolapse (grade III-IV). The 25 patients were then treated with the laparoscopic-modified Wells surgery, with the addition of PPH in 19 cases with rectocele. Notably, the surgery was uneventful with no significant intraoperative complications. Patient characteristics and surgical status are shown in Table 3. A 12-month telephone follow-up was performed after discharge with fecal imaging being performed 6 months after surgery to evaluate the surgical results. To date, none of the 25 patients experienced recurrence.

Compared with preoperative defecography, the proportion of patients diagnosed with rectal prolapse after operation decreased from 36% to 0% (*P* < 0.01), the proportion of patients with severe internal rectal prolapse (grade III-IV) also decreased from 64% to 4% (*P* < 0.01), and the number of patients with rectocele decreased from 20 to 7 (*P* < 0.01). In addition, the number of patients with perineal descent decreased from 23 to 9 (*P* < 0.01), as shown in Table 4 and Supplementary Table (available here).

The anorectal angle during defecation decreased from 138.64 ± 14.18° to 132.68 ± 11.75° after the operation (*P*=0.014). The perineal descent during defecation was improved from 4.75 ± 1.66 cm preoperatively to 2.78 ± 0.80 cm postoperatively (*P* < 0.01). Moreover, the depth of rectocele was improved from 1.37 ± 0.82 cm preoperatively to 0.51 ± 0.33 cm postoperatively (*P* < 0.01) as shown in Figure 1. The postoperative defecography exhibited satisfactory results as shown in Figure 2.

With regard to postoperative clinical symptoms, the proportion of preoperative obstruction and endless defecation was higher than 60%, and most patients were relieved after surgery (*P* < 0.01), as shown in Table 4. Six patients had clinical symptoms of fecal incontinence before surgery, whereas only two patients still had fecal incontinence after surgery. However, their symptoms had been alleviated. There were four patients with constipation before and after the operation, but it could be relieved by dietary guidance and oral laxation. Furthermore, postoperative satisfaction was high in 18 cases (72%), medium in 5 cases (20%), and low in 2 cases (4%).

## 4. Discussion

Defecography is a cost-effective, widely used, and well-established test for evaluating defecation and pelvic floor disorders. This is because it most closely resembles the actual process and position of the patient's bowel movement and provides qualitative and quantitative information about the defecation process [9]. In this study, 107 patients underwent defecography, of which, 102 patients had abnormal defecography results. The percentage of normal results was about 4.7%, which is different from the 12.5% reported by Agachan et al. [10]. Notably, this difference may be attributed to patient selection. Herein, a rectal finger examination was performed at the time of patient admission and then the rectal palpation findings, such as rectal mucosal overlap and anterior rectal void, were combined with clinical symptoms, such as defecation obstruction and incomplete defecation, before recommending defecography to patients, which may explain the high percentage of patients with abnormal imaging results in our examination.

Results showed that there was a higher prevalence of severe internal rectal prolapse in female patients than in male patients, and a significantly higher proportion of combined rectocele and perineal descent in females than in male patients, which is consistent with a previous study [3]. In women, the anterior rectal wall is supported by the rectovaginal septum. However, due to obstetric injury and menopause, the rectovaginal septum of women is relaxed, and the anterior rectal wall tends to protrude forward to form an anterior rectal protrusion. Given that the pelvic floor of women is responsible for the functions of childbirth, intercourse, and defecation, the degree of perineal descent is generally more severe in women than in men with age and history of defecation difficulties [11]. Nevertheless, although the prevalence of rectal prolapse was higher in women than in men, there was no significant difference between the two groups, which is inconsistent with some reports [12]. Notably, this result may be attributed to the small sample size.

With regard to selecting patients for surgery, a large proportion of our outpatients, about 56%, had rectal prolapse and severe internal rectal prolapse. A high percentage of this group of patients also complained of feeling obstruction during defecation. Among them, 25 patients with severe clinical symptoms were treated with a laparoscopic-modified Wells procedure, followed by re-examination using defecography 6 months after the procedure. A comparison of preoperative fecal imaging with postoperative fecal imaging found that most patients benefited from the surgery. Specifically, most patients with a preoperative diagnosis of rectal prolapse and severe internal rectal prolapse improved to no prolapse and mild endorectal prolapse after surgery. Only one patient with a preoperative diagnosis of rectal prolapse still showed severe endorectal prolapse on postoperative fecal imaging, but the patient's clinical symptoms were significantly improved compared to those before surgery. A previous study suggested that correction of internal rectal prolapse can significantly relieve the feeling of bowel obstruction triggered by the accumulation of rectal mucosa and muscularis [13], which was confirmed in this study. It has also been suggested that there is a linear relationship between the severity of fecal incontinence and the grade of endorectal prolapse. Specifically, as the grade of internal rectal prolapse increases, inappropriate excitation of the anorectum inhibition reflex predisposes to urge fecal incontinence [14]. At follow-up, despite there being no significant difference in the number of patients with fecal incontinence, the patients received varying degrees of symptomatic relief.

Preoperative fecal imaging showed a combination of rectocele in 20 patients, 16 of whom complained of incomplete defecation. Our results suggested that the sensation of incomplete defecation was mainly caused by an anterior rectal protrusion. It should be noted that patients with rectocele are unable to expel the fecal masses accumulated in the anterior rectum during defecation and the fecal masses return to the rectum after defecation stops, which causes the patient to feel incomplete defecation and ultimately results in more frequent and excessive straining. This may further aggravate rectal prolapse and endorectal prolapse, thereby resulting in a vicious cycle. Considering that the modified Wells procedure does not contribute to the improvement of rectal prolapse, PPH can not only treat rectocele but can also contribute to the improvement of endorectal prolapse. Regadas et al. reported that they successfully treated eight patients with defecation disorders due to rectocele combined with mucosal prolapse using PPH [15]. PPH can circumferentially remove the prolapsed and redundant rectal mucosa, and aseptic inflammation formed by the anastomotic staple, and fixe the rectal mucosa in the muscular layer of the rectal wall such that the anterior rectal wall becomes a taut interface and no longer produces anterior protrusion, thereby relieving the feeling of incomplete defecation caused by anterior rectal protrusion. Yang et al. achieved better surgical results by using laparoscopic integral pelvic floor/ligament repair combined with PPH to treat internal rectal prolapse [16]. Herein, 19 of the 20 patients with combined rectocele underwent PPH, which resulted in reduction of the number of patients showing postoperative rectal prolapse to seven. At the same time, the symptoms of patients who had a feeling of incomplete defecation before the operation were significantly improved.

Furthermore, the number of patients with perineal descent decreased from 23 preoperatively to nine postoperatively. The causes of perineal descent are complex and are associated with pelvic floor muscle laxity and prolapsed rectal compression. Madbouly et al. reported that the laparoscopic modified Wells procedure improved the degree of perineal descent in patients [17]. The same conclusion was found in this study after comparing the preoperative and postoperative defecography results.

It has previously been reported that preserving the lateral rectal ligament during rectal prolapse surgery avoids damaging the parasympathetic supply to the rectum as well as the vascular supply, thereby reducing the possibility of postoperative constipation without increasing the risk of prolapse recurrence [18]. In this study, the collateral ligament was not cut intraoperatively, and there was no significant increase in the number of patients with postoperative constipation. Similar to the study by Hashida et al., we performed the Wells procedure from the right side of the rectum. Compared to the left-sided approach, the right-sided approach allows for accurate access to the posterior rectal space with more distinct anatomical landmarks. Therefore, it is possible to perform the procedure with a direct view of the ureter and other vital organs, which is safer [19]. The use of glue for patch fixation in ventral mesh rectopexy was reported to be safe, according to Silveira et al. [20]. Thus, we also used a synthetic surgical glue in sacral fixation of the patch, which served as a modified aspect of our laparoscopic procedure. It is worth mentioning that there was no significant glue- and patch-related discomfort during postoperative follow-up and excretion imaging tests.

Defecography is very helpful in the detection of rectal prolapse and has both economic and social benefits. Moreover, rectal prolapse and internal rectal prolapse are common diseases in general surgery clinics and have been studied for many years. However, there are only few studies on the laparoscopic-modified Wells procedure that are conducted in China. Considering the existence of ethnic differences, data from foreign research are limited in guiding Chinese studies. Therefore, this study enriches the domestic research in this field and will aid in introducing and promoting this procedure. However, this study also had some limitations. First, given that this was a single-center retrospective study, the findings may not be generalizable to all patients with rectal prolapse and severe endorectal prolapse. Second, the disease is still underappreciated, and thus patients are generally not willing to undergo surgery, which explains the insufficient sample size. Therefore, future studies and follow-ups on this disease should be conducted in large multicenter samples over a longer period of time.

## 5. Conclusion

This study has proved that defecography can evaluate local functional and morphological changes in the anorectal region and provide imaging data for reference in the diagnosis and treatment of rectal prolapse and internal rectal prolapse. Moreover, the treatment effect of the laparoscopic-modified Wells procedure can be evaluated postoperatively through combining with clinical symptoms.

## Figures and Tables

**Figure 1:** (a) Anorectal angle during defecation between preoperative and postoperative (*P*=0.014). (b) Depth of perineal descent during defecation between preoperative and postoperative (*P* < 0.01). (c) Depth of rectocele between preoperative and postoperative (*P* < 0.01). Significance was estimated using paired *t*-test.

**Figure 2:** (a) Preoperative defecation imaging of a patient with combined severe rectocele. (b) Representative picture of patients after surgery.

**Table 1:** Radiographic findings of defecography in 107 patients.

Parameters	Male *n* = 44	Female *n* = 63	*P* value
Oxford radiological grading			<0.01
No rectal prolapse	23 (52.27)	12 (19.05)	
Internal rectal Prolapse (I-II)	4 (9.09)	8 (12.70)	
Internal rectal Prolapse (III-IV)	11 (25)	28 (44.44)	
Rectal prolapse (V)	6 (13.64)	15 (23.81)	

Perineal descent			<0.01
Combine	14 (31.82)	46 (73.02)	
Not combine	30 (68.18)	17 (26.98)	

Rectocele			<0.01
Combine	13 (29.55)	51 (80.95)	
Not combine	31 (70.45)	12 (19.05)	

Spastic pelvic floor syndrome			0.11
Combine	10 (22.73)	7 (11.11)	
Not combine	34 (77.27)	56 (88.89)	

Colon redundancy			0.75
Combine	12 (27.27)	19 (30.16)	
Not combine	32 (72.73)	44 (69.84)	

Sacrorectal separation			0.51^a^
Combine	0 (0)	2 (3.17)	
Not combine	44 (100)	61 (96.83)	

Significance was estimated using chi-square test. ^a^ Significance was estimated using Fisher's exact test.

**Table 2:** Relationship between different levels of Oxford grading and comorbidity.

Parameters	Oxford grading (I-II, *n* = 12)	Oxford grading (III–V, *n* = 60)	*P* value
Perineal descent			
Combine	5 (41.67)	53 (88.33)	<0.01
Not combine	7 (58.33)	7 (11.67)	

Rectocele			
Combine	7 (58.33)	46 (76.67)	0.34
Not combine	5 (41.67)	14 (23.33)	

Colon redundancy			
Combine	4 (33.33)	18 (0.3)	1
Not combine	8 (66.67)	42 (0.7)	

Spastic pelvic floor syndrome			
Combine	6 (50)	2 (3.33)	<0.01
Not combine	6 (50)	58 (96.6)	

Significance was estimated using chi-square test with correction for continuity.

**Table 3:** Basic information of patients undergoing surgery (*n* = 25).

Parameters	Patient information
Gender (male/female)	9/16
Age (*y*, $\bar{x}\pm s$)	57.8 ± 10.06
Disease course (*y*, $\bar{x}\pm s$)	6.24 ± 2.67
Add PPH procedure [*n* (%)]	19 (76)
Operation time (min, $\bar{x}\pm s$)	163.8 ± 45.68
Blood loss (ml, $\bar{x}\pm s$)	35.6 ± 10.52
Duration of stay (d, $\bar{x}\pm s$)	12.64 ± 3.44
Exhaust time after surgery (d, $\bar{x}\pm s$)	2.12 ± 0.71
First defecation time after surgery (d, $\bar{x}\pm s$)	4.24 ± 0.81

**Table 4:** Preoperative and postoperative defecography and clinical symptoms (*n* = 25).

Parameters	Preoperative	Postoperative	*P* value
Oxford radiological grading			<0.01
No rectal prolapse	0 (0)	18 (72)	
Internal rectal prolapse (I-II)	0 (0)	6 (24)	
Internal rectal prolapse (III-IV)	16 (64)	1 (4)	
Rectal prolapse (V)	9 (36)	0 (0)	

Perineal descent			<0.01
Combine	23 (92)	9 (36)	
Not combine	2 (8)	16 (64)	

Rectocele			<0.01
Combine	20 (80)	7 (28)	
Not combine	5 (20)	18 (72)	

Sense of obstruction			<0.01
Combine	18 (72)	4 (16)	
Not combine	7 (28)	21 (84)	

Sense of endless defecation			<0.01
Combine	16 (64)	6 (24)	
Not combine	9 (36)	19 (76)	

Constipation			1
Combine	4 (16)	4 (16)	
Not combine	21 (84)	21 (84)	

Incontinence			0.125
Combine	6 (24)	2 (8)	
Not combine	19 (76)	23 (92)	

Significance was estimated using McNemar's test.

## Data Availability

The simulation experiment data used to support the findings of this study are available from the corresponding author upon request.

## Supplementary Materials

Supplementary Materials Supplementary Table: Preoperative and Postoperative Oxford Radiological Grading.
